This article has been retracted.

# Biorational Control of *Callosobruchus maculatus* (Coleoptera: Buchidae) in Stored Grains with Botanical Extracts

**DOI:** 10.1155/2022/3443578

**Published:** 2022-08-29

**Authors:** Rasheed Akbar, Imtiaz Ali Khan, Brekhna Faheem, Rashid Azad, Maid Zaman, Rubab Altaf, Amjad Usman, Muhammad Fawad, Abid Farid, Ahmad Ur Rahman Saljoqi, Asad Syed, Ali H. Bahkali, Abdallah M. Elgorban, Jawad Ali Shah, Abdul Qayyum

**Affiliations:** ^1^Department of Entomology, The University of Haripur, Haripur 22620, Pakistan; ^2^Department of Entomology, The University of Agriculture, Peshawar, Pakistan; ^3^Department of Zoology, Abdul Wali Khan University, Mardan, Pakistan; ^4^Department of Environmental Sciences, The University of Haripur, Haripur 22620, Pakistan; ^5^Department of Plant Protection, The University of Agriculture, Peshawar, Pakistan; ^6^Department of Botany and Microbiology, College of Science, King Saud University, P.O. 2455, Riyadh 11451, Saudi Arabia; ^7^Department of Plant Protection, Faculty of Agrobiology Food & Natural Resources, Czech University of life Sciences, Prague, Czech Republic; ^8^Department of Agronomy, The University of Haripur, Haripur 22620, Pakistan

## Abstract

Globally, around 2000 plant species are used against pest control. The utilization of botanicals is considered the most economic and biodegradable methods for the control of stored grains pests. Therefore, the current study was carried out to investigate the repellency potential of five botanicals against *Callosbruchus maculatus* F. in Haripur, Pakistan. The concentrations of *Azadirachta indica* L., *Nicotiana tabacum* L., *Melia azedarach* L., *Nicotiana rustica* L., and *Thuja orientalis* L. were, i.e., 0.5, 1.0, 1.5, 2.0, 2.5, and 3.0% in four replicates to establish contact effects. The data were recorded after 1, 2, 3, 6, 24, 48, 72, and 96 hours. The repellency effect of these plant species against *C. maculatus* were increased in both the time- and dose-dependent manner, and highest effect was observed at 72 h. In addition, the repellency effect was 91% for *A. indica* (class: V), 86% *M. azedarach*, 82%, *N. tabacum* (class: V), 79% *N. rustica* (class: IV), and 75% *T. orientalis* (class: IV) at 3% concentration against *C. maculatus*. Furthermore, following 96 hours' exposure to treatment the sensitivity response of insects decreases as the time interval increases, i.e., 86% *A. indica* (class: V) was followed by 71% *M. azedarach* (class: IV), 65% *N. tabacum* (class: IV), 61% *N. rustica* (class: IV), and *T. orientalis* 57% (class: III) repellency at highest concentration of 3%. The current study concluded that *A. indica* and *M. azedarach* can be incorporated for the management of *C. maculatus* and these plant species might be helpful in the productions of new biopesticides.

## 1. Introduction

The practice of using plant extracts as biopesticides or medicines is well known [1]. As many as 2000 plant species are in use globally in the control of insect pests. Local people adopt more economic and biodegradable method used as different plant part extracts as pesticides against stored products [2]. However, the effectiveness or use of biopesticide increases as pest management in field and stored product pests [3].

Among the stored products, insect pests, the Genus *Callosbruchus* causes annual losses to different stored products including 30% in Mung bean, 20% in pigeon pea and 15% in chick pea [4]. About 2.5-3 million tons of stored grains are lost annually due to *C. maculatus* [5]. The Bruchid beetle, *C. maculatus* F. (Coleoptera: Bruchidae), is a cosmopolitan pest attack on economically important legumes such as mung bean, lentil, black gram, and cow peas [6].

This beetle damages the pulses both quantitatively and qualitatively which then become unfit for consumption [7]. *C. maculatus* breed from March to November and maximum damage is caused from February to August when all the developmental stages are present [8]. It is reported that farmer uses highly toxic insecticides to protect their stored commodities including mung bean. The use of chemical insecticides which have known side effects including handling hazards, toxic residues, and development of insecticide resistance [9]. Therefore, insecticides having toxic residues should be discouraged for the control of insect pests [10]. Due to injudicious use of insecticides, most of the stored product pests showed resistance against synthetic insecticides [11].

It is necessary to investigate alternative sources for the management of stored insect pests [12]. For the control of insect pests in storage, there is limited information regarding the utilization of plant products. Overuse of insecticides creates resistance in pest and has a harmful impact on the environment. Therefore, alternative strategies for the management of pests should be adopted [13]. The plant extracts not only environmental friendly but also social acceptable and easily available for local store keeper, farmers, and the people whose business is related with stored commodities. Keeping in view the importance of botanicals pesticides, the present studies were conducted with the aims to find out repellency response of *C*. *maculatus* against different plant extracts.

## 2. Material and Methods

The experiment was laid out in completely randomized design (CRD) with factorial arrangement having five treatments each with four replications. The leaves and fruits of five selected plants viz. *A. indica*, *M. azedarach*, *N. rustica*, *N. tabacum*, and *T. orientalis* were collected from different locations of district Swabi, Khyber-Pakhtunkhwa Pakistan (as shown in Table 1 and Figure 1).

### 2.1. Collection and Establishment of Stock Culture Insects

*C. maculatus* were collected from infested godowns at District Swabi. The collected *C. maculatus* were then brought to Entomological Laboratory, Department of Entomology, the University of Haripur, and released in a glass jar having mung bean as favorite food medium; the jars were covered with muslin cloth and kept in the lab at 30°C and 60 ± 5% RH [9].

### 2.2. Preparation of Plant Aqueous Extract

Six concentrations of all the selected 5 botanicals were prepared according to the methods adopted by [14]. Leaves and fruits were placed in distilled water for the duration of 48 hr. 0.25, 0.50, 0.75, 1.00, 1.25, and 1.50 g of each botanicals (different parts) were directly diluted in 50 ml of distilled water to make 0.5, 1, 1.5, 2 2.5 and 3% (*w*/*v*) solution. Each concentration was prepared separately [9].

### 2.3. Phytochemical Screening of Selected Plant Aqueous Extracts

The standard solution of 200 ml extracts was prepared by mixture of selected plant extract and distilled water [15]. The extracts were subjected for phytochemical for the following standard methods.

#### 2.3.1. Extraction Procedure

Maceration: For maceration (for fluid extract), whole or coarsely powdered plant drug was kept in contact with the solvent in a stopper container for a defined period with frequent agitation until soluble matter is dissolved [16].

#### 2.3.2. Tests for Alkaloid Wegener's tests

Extracts of the test plants were dissolved individually in dilute hydrochloric acid 1.5% and filtered with Whatman No. 1 filter paper by the treatment filtrates with few drops of iodine in 2 to 3 drops of potassium iodide. The presence of brown reddish precipitates that pointed out the presence of alkaloids in the samples [17].

#### 2.3.3. Tests for Phenols

In ferric chloride test, for the screening of phenol plant aqueous extracts, the phenol plant aqueous extracts were treated with 3-4 drops of ferric chloride solution. The appearance of bluish black color indicated the presence of phenols [18].

#### 2.3.4. Tests for Phytosterols: Salkowski's Test

The test plant aqueous extracts were treated with chloroform and filtered with Whatman no. 1 filter paper. Few drops of concentrated sulphuric acid were added and then vertexed it and allowed to stand for some time. The golden yellow color indicated the presence of phytosterol [18].

#### 2.3.5. Tests for Diterpenes

To observe the presence of diterpenes, the plant aqueous extracts were treated with 3-4 drops of copper acetate solution. Formation of emerald green color indicated the presence of diterpenes [18].

#### 2.3.6. Tests for Saponins

For dilution about 2 ml of plant aqueous extracts were taken in test tube, in distilled water and vortexed it for 5 minutes. Foam produced and persisted for ten minutes indicated the presence of saponins [17].

#### 2.3.7. Tests for Flavonoids

In the alkaline reagent test, for the presence of flavonoids, the plant aqueous extracts were treated with 2-3 drops of lead acetate solutions. The formation of intense yellow color, which becomes colorless on addition of dilute acid, indicated the presence of flavonoids [19].

### 2.4. Bioassay of C. maculatus Adults

The repellency effect of tested botanicals used against the beetles was assessed by using the area preference method [9]. In bioassays, 6 concentrations viz. 0.5, 1, 1.5, 2, 2.5, and 3% of aqueous extracts were used. Whatman No.1 filter paper was equally divided into 2 halves (about 7.2 cm diameter). First half portion of each filter paper was treated with the extract by using micropipette, and the 2nd half portion of filter paper was treated with distilled water as a control. Each filter paper was air dried for about 30 minutes, till complete evaporation of solvent. The filter paper was then pasted length wise, edge wise with the help of masking tape and kept at the bottom of 16 cm diameter Petri dishes. Ten pairs of freshly emerged adult beetles (total of 20 per dish) were released at the center of the test arena in the Petri dishes and covered with muslin cloth and kept in an incubator at 27 ± 2°C and 65 ± 5% relative humidity. Total numbers of insects residing on treated and untreated portions of filter paper were counted after 1, 2, 3, 6, 24, 48, 72, and 96 hours, and percent repellency (PR) was calculated by using the formula adopted by [20]

(1) $$\begin{array}{c} \text{PR}=\left[\frac{Nc-Nt}{Nc}\right]\times 100, \end{array}$$

where *Nc* is the no. of insects counted in control and *Nt* is the no. of insects counted in treated.

The botanicals were then categorized into different classes (as shown in Table 2), [21].

### 2.5. Statistical Analysis

The recorded data were subjected to analysis of variance (ANOVA) with two factors CRD (complete randomized design), and means were separated by using the least significant difference (LSD) test at 5% level of probability. Statistical analyses were carried out using STATISTIX 8.1 [22].

## 3. Results

### 3.1. Screening of Aqueous Extracts of Plants for Phytochemical Constituents

In this experiment, phytochemical constituents of five plant species were determined from their crude extracts (as shown in Table 3). It was clear from the results that all the phytochemical constituents were present in *M. azedarach*, with both phytosterol and phenol in moderate amount while the rest of phytochemicals were present in lower quantities. *A. indica* also exhibited all the phytochemicals in high quantities. Moreover, in *N. tabacum* all the phytochemicals were present, whereas diterpenes and phenols were present in high amount and the others in moderate quantities. In *N. rustica*, saponins were not present while, rest in low quantities. In *T. orientalis*, all the phytochemicals were present in low quantities.

### 3.2. Repellency

The settling response of *C. maculatus* was significantly (*P* < 0.05) affected by concentration. The adults of *C. maculatus* preferred the untreated arena (control) as compared with treated arena. The preference response of tested insects significantly declined with the increases in concentrations of extracts. The repellency of five different botanicals against *C. maculatus* were studied under controlled laboratory conditions, and result revealed different trends in different parameters which are explained as follows.

#### 3.2.1. Mean Percent Repellency of C. maculatus after 1 h Exposure Period

After one hour of exposure, highest repellency of *C. maculatus* was observed with *A. indica* (53.75 ± 4.26) (*df* = 5, *P* < 0.05, *F* = 34.38) which show class III repellency, while the lowest was recorded with *T. orientalis* (32.25 ± 0.75) which show class II repellency. An increasing trend in repellency was observed with the increase in concentration of botanicals (Figure 2).

#### 3.2.2. Mean Percent Repellency of C. maculatus after 2 h Exposure Period

The repellency of tested botanical against *C. maculatus* after two hours of exposure. *A. indica* showed the highest repellency (57.5 ± 3.22) against *C. maculatus*, and the lowest repellency was observed with *T. orientalis* (41.25 ± 3.75) (*df* = 5; *P* < 0.05; *F* = 34.38) (Figure 3).

#### 3.2.3. Mean Percent Repellency of C. maculatus after 3 h Exposure Period

Result showed the highest repellency of *C. maculatus* against *A. indica* (60 ± 2.04) at 3% concentration, while the lowest repellency was observed against *T. orientalis* (51.5 ± 3.09) (*df* = 5; *P* < 0.05; *F* = 49.98) after the exposure period of 3 hours (Figure 4).

#### 3.2.4. Mean Percent Repellency of C. maculatus after 6 h Exposure Period

Results described the repellency of tested botanical insecticides against *C. maculatus* (*df* = 5; *P* < 0.05; *F* = 49.33). At 3% concentration after 6 hours of exposure, highest repellency (class IV repellency) was recorded in *A. indica* (66 ± 3.7). In comparison, the lowest repellency (class III repellency) was observed in *T. orientalis* (51.25 ± 2.39) (Figure 5).

#### 3.2.5. Mean Percent Repellency of C. maculatus after 24 h Exposure Period

After 24 hours of exposure at 3% concentration (*df* = 5; *P* < 0.05; *F* = 54.07), highest repellency was observed in *A. indica* (72.5 ± 2.5) and the lowest repellency was observed in *T. orientalis* (60.25 ± 2.25) (Figure 6).

#### 3.2.6. Mean Percent Repellency of C. maculatus after 48 h Exposure Period

After 48 hours of exposure, the repellency effect of different concentration of selected plant extract presented (Figure 7) (*df* = 5; *P* < 0.05; *F* = 109.38). Results revealed the highest repellency (class V repellency) at 3% concentration in *A. indica* (85 ± 2.04) while the lowest repellency was observed in *T. orientalis* (70 ± 2.04) (class IV repellency).

#### 3.2.7. Mean Percent Repellency of C. maculatus after 72 h Exposure Period

After 72 hours of exposure (*df* = 5; *P* < 0.05; *F* = 104.80), *A. indica* (91.25 ± 1.49) showed the highest repellency (class V repellency), while the lowest repellency (class III repellency) was recorded in *T. orientalis* (75 ± 3.53) at 3% concentration (Figure 8).

#### 3.2.8. Mean Percent Repellency of C. maculatus after 96 h Exposure Period

After 96 hours (*df* = 5; *P* < 0.05; *F* = 123.10), the repellency effect of tested plant extract against *C. maculatus* was significantly presented. Decreasing trend in repellency was observed after 72 hours of exposures; however, the highest repellency (class V repellency) was observed in *A. indica* (86.25 ± 1.75) and lowest repellency (class III repellency) was observed in *T. orientalis* (57.5 ± 1.44) at 3% concentration (Figure 9).

## 4. Discussion

Entomologists and pest controllers around the world are using plant-based insecticides increasingly frequently, most likely as a result of public awareness of the risks connected with many chemical pesticides. However, the method of extraction, the section of the plant used, and the type of solvent employed for their extraction all directly or indirectly affect the efficiency of many botanical insecticides [23]. Different solvents' polarities may result in variations in how well they extract the active ingredient found in botanicals. Present experiments based on phytochemicals in five plants species yielded variable results. All the phytochemicals were found in all the five plant species. Some earlier researchers have reported results similar to the current study, such as [24] reported that the aqueous extract of *N. tabacum* leaves tested positive for alkaloids, tannins, flavonoids, steroids, cardiac glycosides, essential oils, resins, and polypeptides. [25] stated that tobacco leaves contain nicotine, as we know that nicotine is an alkaloid which is the most biologically active component of tobacco. Alkaloids, being one of the largest group of phytochemicals in plants have pronounced effect on humans which have led to development of pain killer medication [26]. Moreover, these alkaloids have also been act as insect repellents as mentioned by [27]. According to [28], *A. indica* crude extracts showed the presence of alkaloids, glycosides, flavonoids, saponins, tanins, and phenolic compounds. In the present research, crude extracts of *M. azedarach* indicated high presence of terpiniods, saponins, flavonoids, and phenols. [29] yielded results similar to our findings. According to [30], crude extracts of *M. azedarach* gave phenols, flavonoids, tannins, alkaloids, terpinoids, and saponins.

Outcomes of the present studies are consistent with [31] who also reported the highest repellency of *A. indica* against *T. castaneum*, with decreasing trend with the passage of time. Our results also agreed with some earlier researcher [32, 33] that *A. indica* repels insect and causes them to stop their feeding. Neem extracts contain azadirichtin and salannin that function as insect feeding deterrent. [34, 35] also reported the use of *A. indica* for the control different foliage pests. In case of *M. azedarach*, our results are in agreement with [36] who also reported that the repellency effect of *M. azedarach* decreases after the 72-hour exposure period. Research carried out worldwide during the last three decades have also shown significant repellency effect of the *M. azedarach* for the management of stored product pests [30]. Tobacco (*N. tabacum* and *N. rustica*) is traditionally known as a natural insecticide [37]. In our studies, we observed 82% repellency in *N. tabacum* and 76% in *N. rustica* against *C. maculatus* at 3% concentration. Our results are agreed with [38] who recorded similar repellency trend as in our study (increases repellency at increased concentration of plant extracts. This result also coincides with the findings of [39] who also reported the maximum repellency in *N. tabacum* at high concentration against *T. castaneum.* Nicotiana species contain nicotine which is an alkaloid act as a potent insecticide that bind the acetylcholine receptor and affect the nerve transmission that act as a feeding deterrent. In our study, among the tested botanicals, the lowest repellency was observed in *T. orientalis* against *C. maculatus*. Our results are in contradiction with the findings of [40] who observed high repellency (92%) in *T. orientalis* against *Tribolium confusum.* Difference in results might be due to the different plant parts used for the extraction that have different percentage compositions of the ingredients [41]. The insecticidal constituents of many plant extracts and essential oils are mainly monoterpenoids [42]. Monoterpenoids are typically volatile and rather lipophilic compounds that can penetrate into insects rapidly and interfere with their physiological functions [43]. Due to their high volatility, they have fumigant activity that might be of importance for controlling stored product insects [44]. Studies carried out worldwide during last the three decades have significantly extended our knowledge on botanical pesticides. Many plant-derived natural products active against insect could be produced from locally available raw materials, perhaps in many cases right at the site of usage, so as to be relatively inexpensive [43]. In this study, pure liquid extract of *A. indica* and *M. azedarach* was effective at managing the population of *C. maculatus*. It may therefore be one of the alternative control options in our immediate environment. The natural phytochemicals from Plants have potential being ecofriendly can replace synthetic pesticides for the insect pests [45]. Nevertheless, despite their efficiency, the extracts have no negative impact on the stored pulses. Consequently, these plant extracts may be utilized to help reduce the number of *C. maculatus.*

## 5. Conclusion

It is reported that the utilization of phytochemicals is ecofriendly, socially acceptable, and economically feasible approach for the management and biocontrol of *C. maculatus*. Based on our result, it can be concluded that *A. indica* and *M. azedarach* at all concentration might serves as alternative to insecticides in rural areas of tropic and subtropic region. The promising and effective repellency of these botanicals suggesting that these botanicals as a potential candidate agent against the *C. maculatus* and can be recommended for their integration with other control strategies that will reduced environmental pollution and health hazards problems. Moreover, use of these plant extracts can open new avenue for the management of *C. maculatus.*

## Figures and Tables

**Figure 1:** Location from which plant species collected during 2021.

**Figure 2:** Mean percent repellency of *C. maculatus* after 1-hour exposure period treated with six different concentrations of crude extracts of five plant species.

**Figure 3:** Mean percent repellency of *C. maculatus* after 2-hour exposure period treated with six different concentrations of crude extracts of five plant species.

**Figure 4:** Mean percent repellency of *C. maculatus* after 3-hour exposure period treated with six different concentrations of crude extracts of five plant species.

**Figure 5:** Mean percent repellency of *C. maculatus* after 6-hour exposure period treated with six different concentrations of crude extracts of five plant species.

**Figure 6:** Mean percent repellency of *C. maculatus* after 24-hour exposure period treated with six different concentrations of crude extracts of five plant species.

**Figure 7:** Mean percent repellency of *C. maculatus* after 48-hour exposure period treated with six different concentrations of crude extracts of five plant species.

**Figure 8:** Mean percent repellency of *C. maculatus* after 72-hour exposure period treated with six different concentrations of crude extracts of five plant species.

**Figure 9:** Mean percent repellency of *C. maculatus* after 96-hour exposure period treated with six different concentrations of crude extracts of five plant species.

**Table 1:** List of plant species and plant parts used in the experiment with *C. maculatus* during 2021.

Sr. no.	Common name	Botanical name	Family	Part used
1	Neem	*Azadirachta indica*	Meliaceae	Seed
2	Bakion	*Melia azedarach*	Meliaceae	Fruit
3	White Patta	*Nicotiana rustica*	Solanaceae	Leave
4	Virginia tobacco	*Nicotiana tabacum*	Solanaceae	Leave
5	Chinese arborvitae	*Thuja orientalis*	Cupressaceae	Fruit

**Table 2:** Repellency classes according to McDonald et al. [21].

Sr. no.	Class	&*R*1
1	0	>0.01-0.1
2	I	0.1-20
3	II	20.1-40
3	III	40.1-60
4	IV	60.1-80
5	V	80.1-100

1%*R*: percentage of repellency rate.

**Table 3:** Phytochemical composition of crude extracts of five plant species during 2021.

Plant species	Phytochemical constituents of five plant species					
	Alkaloids	Flavonoids	Saponins	Diterpenes	Phytosterol	Phenols
*A. indica*	+++	+++	++	++	+++	+++
*N. tabacum*	++	++	++	+++	++	+++
*M. azedarach*	+	+	+	+	++	++
*N. rustica*	+	+	—	+	+	+
*T. orientalis*	+	+	+	+	+	+

+++: highly present; ++: moderately present; +: low present; –: not present.

## Data Availability

Data is included in the article.

## Additional Points

*Novelty of the Study*. This laboratory work evaluated the anti-insect potential of local plant species from District Swabi and Haripur, Khyber Pakhtunkhwa of Pakistan, against destructive insect pest of stored grain, i.e., *Callosobruchus maculatus*. Bioassays revealed that water extracts of *A. indica*, *M. azedarach*, *N. rustica*, *N. tabacum*, and *T. orientalis* at various concentrations particularly at 3% and exhibited considerable repellency of insect pest individuals suggesting their biocidal potential against this insect pest.
